RETRACTED

# Analysis of Landscape Ecological Planning Based on the High-Order Multiwavelet Neural Network Algorithm

**DOI:** 10.1155/2021/9420532

**Published:** 2021-07-23

**Authors:** ChuanDong Yu, Nan Du

**Affiliations:** ^1^The Art Design and Public Administration Department, YanTai Vocational College, Yantai 264670, Shandong, China; ^2^Department of Radio and Television Directing, Ludong University, Yantai 264000, Shandong, China

## Abstract

Landscape architecture has both natural and social properties, which is the embodiment of people protecting the natural environment. Since the industrial revolution, the modern industry has developed rapidly. It has increased the living standard of people and consumed a lot of natural resources such as forest and energy. The ecological environment has been greatly damaged, and the landscape of gardens has been affected. Therefore, it is of great significance to find a method to evaluate the landscape ecology and plan the landscape ecology. This paper proposes a new high-order wavelet neural network algorithm combining wavelet analysis and artificial neural network. A model of ecological evaluation of landscape based on high-order wavelet neural network algorithm is proposed to evaluate the landscape ecology and provide reference data for the ecological planning of the landscape. The results show that the training times of the wavelet neural network to achieve the target accuracy are 3600 times less than those of the BP neural network. The MSE and MAE of the WNN are 0.0639 and 0.1501, respectively. The average error of the model to the comprehensive evaluation index of the landscape ecology is 0.005. The accuracy of the model to evaluate the sustainability of landscape land resources is 98.67%. The above results show that the model based on the wavelet neural network can effectively and accurately complete the evaluation of landscape ecology and then provide a decision-making basis for landscape ecological planning, which is of high practicability.

## 1. Introduction

The development of the chemical industry leads to the deterioration of the ecological environment, which seriously threatens the survival of human beings. Therefore, it is necessary to take early measures to maintain the ecological environment [1]. Landscape refers to the interaction and dynamic coordination among multiple ecosystems in a region. The research and application of landscape dynamic changes and ecological principles will contribute to the development of traditional ecology, provide a new idea for the protection of the ecological environment, and then make humans out of the current dilemma of ecological environment problems [2]. The basic form of landscape can be divided into soft landscape and hard landscape: soft refers to the natural landscape, and hard generally refers to the landscape. Landscape has both natural and social attributes, which is a special landscape dominated by human activities [3]. The ecological planning of landscape refers to the planning measures taken to ensure the ecological balance of landscape based on the principles of ecology and the laws of society and nature. Therefore, the ecological planning of landscape can improve the status of the ecological environment, ensure the good development of the ecological environment, and also make people feel the importance of environmental protection [4]. A high-order wavelet neural network (WNN) algorithm combining wavelet analysis and artificial neural network is proposed, and a landscape ecological evaluation model based on high-order wavelet neural network algorithm is constructed, so as to evaluate the landscape ecology and provide reference data for landscape ecological planning.

RETRACTED

Ouma et al. [5] established models by using the WNN and long short-term memory network (LSTM) neural network, respectively, to predict the trend of rainfall and runoff in the Nzoia River Basin. The results show that both models are competent for this function. Dhibi and Ben Amar [6] proposed a new method based on the multimother wavelet neural network (MMWNN) structure optimized by genetic algorithm to deal with Laplacian boundary deformation, and compared with the method based on LM algorithm, the results show that the processing speed and accuracy of the new method are better than those based on LM algorithm. Huang and Chao [7] used ant colony algorithm (ACO) to optimize the wavelet neural network and built the ACO-WNN model to predict the HL and Cl values of residential buildings. Compared with the traditional WNN model, the average absolute errors of HL and Cl predicted by this model decreased by 82.44% and 84.82%, respectively. Alexander et al. [8] built a prediction model based on the genetic algorithm-optimized regression wavelet neural network to predict building energy consumption, which is 22.6% less than the traditional autoregressive moving average error regression model. Tang et al. [9] combined the random forest and wavelet neural network algorithm to establish the RF-WNN model to evaluate the frost resistance of concrete. The results show that the predicted value of the RF-WNN model is very close to the actual value. Hasanzadeh Fereydooni et al. [10] used the wavelet neural network to obtain the expected trajectory of patients based on the sEMG signal and then guided the intelligent control design of the rehabilitation robot.

RETRACTED

Xu et al. [11] used the wavelet neural network to determine the content of soil organic carbon (SOC). The research shows that the WNN model has a certain effect, but the effect is not as good as the SVMR-FDR model. Du et al. [12] combined a whale optimization algorithm (IWA) with the WNN to build the IWA-WNN model to predict urban traffic flow. The research results show that the prediction speed and accuracy of the model are better than those of the traditional WOA-WNN model. Luo et al. [13] established the FO equation of the gyro coupled system, used the fuzzy wavelet neural network (FWNN) with transformation to approximate the unknown function of the system, and studied the dynamic analysis and accelerated optimal stabilization of the fractional-order self-supporting electromechanical seismograph system under the energy mechanism, and the results show that the method is effective. Wu and Huang [14] used fuzzy wavelet neural networks (FWNNS) to estimate the dynamic uncertainty of OMRM and then study the terminal sliding mode control strategy of the omnidirectional mobile robot. The results show that the method is feasible. Tabaraki et al. [15] constructed a principal component-wavelet neural network (PC-WNN) nonlinear model to predict the critical micelle concentration of anionic gemini surfactants. The results show that the prediction performance of this model is better than that of other models.

It can be seen from the above content that there are many research studies on the application of the wavelet neural network, and the application fields are also very wide, but few research studies apply the wavelet neural network to the ecological planning of landscape. Based on the high-order wavelet neural network algorithm, this paper constructs the ecological evaluation model of landscape, makes statistics and analysis on various parameters affecting the landscape ecology, and gives objective and accurate evaluation results, so as to provide a scientific and effective basis for the ecological planning of landscape.

## 2. Landscape Ecological Evaluation Model

### 2.1. Ecological Planning of the Landscape Architecture

The central idea of landscape ecological planning is to protect the ecological environment. Therefore, in the ecological planning of landscape, we need to consider not only the aesthetic value of landscape but also the ecological value of landscape. Therefore, the following principles should be followed in landscape ecological planning.

Principle of sustainability: in landscape planning, we should ensure the long-term practicability of landscape, conform to the law of natural development, and ensure ecological balance; conservation principle: in ecological planning, local climate, environment, and other factors should be taken into account to make the landscape and environment reach a coordinated state, so as to improve the living environment. In addition, renewable resources should be used as much as possible in planning, and resources should be used efficiently and circularly [16]; practical principle: in the planning, the landscape needs to be in line with the reality and formulate the reasonable planning content [17]; economic principle: when carrying out ecological planning, we should try to control the cost and spend the least money to plan the most satisfactory effect. In order to achieve the above effect, we need to obtain the specific parameters of the landscape and make a detailed assessment of the ecological status of the landscape in order to achieve reasonable ecological planning.

RETRACTED

### 2.2. Landscape Ecological Evaluation Based on the WNN Model

The evaluation process of the WNN model on the ecological status of the landscape is shown in Figure 1.

In the above content, the evaluation index system has a great impact on the accuracy of the WNN model in the evaluation of the ecological status of landscape. Therefore, in the investigation and research of landscape, it is necessary to obtain as many parameters as possible that can reflect the ecological status of landscape and process them to ensure the accuracy of the data [18].

## 3. Construction of the Landscape Ecological Evaluation Model

### 3.1. Establishment of the Ecological Evaluation Index System for the Landscape Architecture

Artificial neural network (ANN) is generally used to build the evaluation model for landscape planning. Artificial neural network (ANN) is a kind of network composed of a large number of nodes connected according to different connection ways, which plays an important role in intelligent robots, biology, medicine, and other fields. However, the evaluation model constructed by the artificial neural network is slow in speed and low in accuracy. A high-order multiwavelet neural network algorithm based on wavelet is constructed to evaluate the landscape ecological state [19]. WNN model is a mapping analysis of landscape ecology, as shown in Figure 2.

The premise of the above content is to build the ecological evaluation system of landscape to ensure the accuracy of the model. When selecting evaluation indexes, we need to follow the principles of comprehensiveness, leading factors, scientificity, regionality, and dynamism [20]. In this paper, the comprehensive index method is used to evaluate each comprehensive index of the landscape and then to find the ecological defects of the landscape, so as to better and pertinently complete the ecological planning of landscape. The landscape ecological index is shown in the following formula:

(1) $$\begin{array}{c} P=\overset{m}{\underset{i=1}{\sum }}\overset{n}{\underset{j=1}{\sum }}C_{ij}\cdot w_{j}. \end{array}$$

In formula (1), *P* is the comprehensive evaluation index of landscape ecology, *i* refers to a certain area in the landscape, *j* is an evaluation index, *C*_*ij*_ is the score of some index *j* in the *i* area, and *w*_*j*_ is the weight of the *j* index in the whole landscape ecological status. The corresponding standards of different ecological comprehensive evaluation values are shown in Table 1.

RETRACTED

By using the empirical method and principal component analysis (PCA) to screen the corresponding indicators, three first-level indicators, such as landscape output function (*C*1), landscape threat degree (*C*2), and landscape stability (*C*3), and several second-level indicators are selected, and then the landscape ecological status evaluation index system is established, as shown in Figure 3.

The evaluation index system of landscape ecological status is a set of nonlinear data, and the artificial neural network can well estimate the nonlinear function, so the artificial neural network is used to deal with the evaluation index. The nodes in the artificial neural network are called artificial neurons. Neurons can process information nonlinearly, and the information transmission mode is multiple-input single-output. Their structure is shown in Figure 4.

The relationship between the input and output of the neuron in the artificial neural network is shown in the following formula:

(2) $$\begin{array}{c} \left\{\begin{array}{c} u_{i}=\sum w_{ij}x_{j}+s_{j}-\theta_{i},\\ y_{i}=f\left(u_{i}\right). \end{array}\right. \end{array}$$

In formula (2), *u*_*i*_ is the neuron, *x*_*j*_ is the input variable, *w*_*ij*_ is the connection weight, *s*_*i*_ is the external input control signal, *u*_*i*_ can be controlled, *θ*_*i*_ is the threshold, and *y*_*i*_ is the output value. There are two kinds of learning methods of the artificial neural network, namely, supervised learning and unsupervised learning. In this study, tutored learning method is adopted to speed up the learning speed and accuracy of the neural network.

### 3.2. Construction of the High-Order Multiwavelet Neural Network Model

BP neural network is the most common neural network, which has a wide range of applications in various fields [21]. It can express the nonlinear mapping with high complexity, and the ecological status evaluation model of landscape is to describe the nonlinear mapping relationship between various indicators, so the BP neural network is used as the model [22]. The structure of the BP neural network is shown in Figure 5.

RETRACTED

The neuron activation function of the BP neural network needs to be differentiable at any place, so sigmoid function is selected as the neuron activation function, as shown in the following formula:

(3) $$\begin{array}{c} f\left(x\right)=\frac{1}{1+e^{-x}}. \end{array}$$

The wavelet neural network is formed by integrating the operation method of wavelet analysis into the neural network [23]. Compared with the traditional BP neural network, wavelet neural network has higher approximation accuracy, simpler network structure, and faster convergence speed [16]. For the nonlinear function, the wavelet neural network uses the wavelet to fit the nonlinear function, as shown in the following formula:

(4) $$\begin{array}{c} \hat{y}\left(x\right)=\sum_{i=1}^{n}w_{i}h\left(\frac{\sum_{i=1}^{m}u_{ti}X_{t}\left(i\right)-b_{t}}{a_{t}}\right). \end{array}$$

In formula (4), for a nonlinear function *y*(*t*), the fitting value sequence is expressed as $\hat{y}\left(x\right)$; *u*_*ti*_ is the connection weight between the *t* unit in the middle layer of the BP neural network and the *i* unit in the input layer of the BP neural network, and *w*_*i*_ is the connection weight between the output layer and the *i* unit in the middle layer; *b*_*t*_ is the translation factor of the wavelet basis, and *a*_*t*_ is the expansion factor of the wavelet basis; *n* is the number of wavelet bases. In order to minimize the error of $\hat{y}\left(x\right)$, the minimum mean square error energy function is used to optimize it. The minimum mean square error energy function is shown in the following formula:

(5) $$\begin{array}{c} E=\frac{1}{2}\sum_{t=1}^{N}{\left[y\left(x\right)-\hat{y}\left(x\right)\right]}^{2}. \end{array}$$

The essence of formula (5) to optimize $\hat{y}\left(x\right)$ is to optimize its network parameters. The steps are as follows: initialize *a*_*t*_, *b*_*t*_, *u*_*ti*_, and *w*_*i*_; input learning sample *x*_*i*_(*i*) and expected output $\hat{y}\left(x\right)$; make wavelet neural network self-learning; obtain the instantaneous gradient vector; and make error backpropagation, as shown in the following formula:

(6) $$\begin{array}{c} \left\{\begin{array}{c} △w_{t}^{\text{new}}=-\eta \frac{\partial E}{\partial w_{t}^{\text{old}}}+a△w_{t}^{\text{old}},\\ △a_{t}^{\text{new}}=-\eta \frac{\partial E}{\partial a_{t}^{\text{old}}}+a△a_{t}^{\text{old}},\\ △b_{t}^{\text{new}}=-\eta \frac{\partial E}{\partial b_{t}^{\text{old}}}+a△b_{t}^{\text{old}},\\ △u_{t}^{\text{new}}=-\eta \frac{\partial E}{\partial u_{t}^{\text{old}}}+a△u_{t}^{\text{old}}. \end{array}\right. \end{array}$$

According to the feedback result of formula (6), the network parameters of the wavelet neural network are modified. For the expansion factor of the wavelet basis, the modification method is shown in the following formula:

(7) $$\begin{array}{c} a_{t}^{\text{new}}=a_{t}^{\text{old}}-△a_{t}^{\text{old}}. \end{array}$$

For the translation factor of the wavelet basis, the modification method is shown in the following formula:

(8) $$\begin{array}{c} b_{t}^{\text{new}}=b_{t}^{\text{old}}-△b_{t}^{\text{old}}. \end{array}$$

For the connection weight between the middle layer and the input layer, the modification method is shown in the following formula:

(9) $$\begin{array}{c} u_{ti}^{\text{new}}=u_{ti}^{\text{old}}-△u_{ti}^{\text{old}}. \end{array}$$

For the connection weight between the output layer and the middle layer, the modification method is shown in the following formula:

(10) $$\begin{array}{c} w_{t}^{\text{new}}=w_{t}^{\text{old}}-△w_{t}^{\text{old}}. \end{array}$$

If it is less than the preset value, the wavelet neural network stops learning; otherwise, continue to input samples and expected output values, and continue to learn. The principle of the wavelet neural network to evaluate the ecological status of landscape is as follows: wavelet basis is used as the hidden layer incentive function of the ANN, the value describing the characteristics of the evaluation object is used as the input vector, and the known evaluation value is used as the output vector. After training with a large number of sample data, the wavelet neural network has enough evaluation experience and reasoning mechanism. The ecological status of landscape can be comprehensively evaluated. The structure of the WNN is shown in Figure 6.

RETRACTED

The basic model of the wavelet transform is shown in the following formula:

(11) $$\begin{array}{c} W_{f}\left(a,b\right)=\int_{-\infty }^{+\infty }f\left(t\right)h\left(a,b,t\right)\text{d}t. \end{array}$$

In formula (11), *f*(*t*) is a function with compact support, and *h*(*a*, *b*, *t*) is a wavelet and satisfies the following formula:

(12) $$\begin{array}{c} h\left(a,b,t\right)=\frac{1}{\sqrt{\left|a\right|}}h\left(\frac{t-b}{a}\right). \end{array}$$

In formula (12), $\left(1/\sqrt{\left|a\right|}\right)$ is the normalized coefficient, and *h*(*t*) is the mother wavelet. In order to train the comprehensive evaluation model of landscape ecological status based on the WNN, we need to obtain the corresponding network parameters *W*_*k*_, *b*_*k*_, and *a*_*k*_ and optimize them with the following formula:

(13) $$\begin{array}{c} E=\frac{1}{2}\sum_{s=1}^{s}\sum_{n=1}^{n}{\left(d_{ns}-v_{ns}\right)}^{2}. \end{array}$$

In formula (13), *d*_*ns*_ represents the desired classified output of the input signal *f*_*n*_(*t*); *v*_*ns*_ is the output value of the neural network under the current network parameters. There are many types of fundamental wavelets in the wavelet neural network. Cosine-modulated Gaussian wave is commonly used in the research, and its expression is shown in the following formula:

(14) $$\begin{array}{c} \psi \left(t\right)=\cos\left(1.75t\right)\exp\left(-\frac{t^{2}}{2}\right), \end{array}$$

(15) $$\begin{array}{c} v_{ns}=\delta \left[\sum_{k=1}^{k}W_{k}\sum_{t=1}^{t}f_{n}\left(t\right)\psi \left(\frac{t-b_{k}}{a_{k}}\right)\right]. \end{array}$$

After obtaining the current output value of the model, the gradient vector is calculated, and the error is backpropagated to obtain the modified network parameters. When the error function value is less than the preset value, the model will end learning and obtain the evaluation parameter value of the landscape ecological status; otherwise, continue learning.

RETRACTED

## 4. Performance Analysis of the Ecological Evaluation Model of the Landscape

### 4.1. Performance Analysis of the Wavelet Neural Network

In order to evaluate the ecological status of landscape, the ecological evaluation model of landscape based on the wavelet neural network was constructed. In order to verify the performance of the wavelet neural network, the wavelet neural network and traditional BP neural network (BPNN) were used to build the landscape ecological evaluation model, the same sample dataset was used to train the two models, and the training time of the two models was compared. The training results are shown in Figure 7.

As can be seen from Figure 7, the wavelet neural network needs 1700 times of training to achieve the target accuracy (0.0001), while the BP neural network needs 5300 times of training to achieve the target accuracy, 3600 times more than the wavelet neural network. WNN model and BPNN model are used to evaluate the ecological value of a landscape, and the evaluation results are compared with the real value. The error of the evaluation results of the two models is expressed by mean square error (MSE) and mean absolute error (MAE). The results are shown in Table 2.

As can be seen from Table 2, the MSE of the WNN and BPNN is 0.0639 and 5.4072, respectively, which is 5.3433 times higher than the WNN. The MAE of the WNN is 0.1501 and BPNN is 1.1330, which is 0.9829 times higher than the WNN. Mean square error (MSE) and mean absolute error (MAE) were used to verify the landscape diversity assessment results of a landscape by the WNN and BPNN, as shown in Table 3.

As can be seen from Table 3, the MSE of landscape diversity assessment results of the WNN and BPNN is 0.0597 and 5.0801, respectively, which is 5.0204 times higher than the WNN. The MAE of the WNN and BPNN was 0.1150 and 0.9914, respectively, which was 0.8764 times higher than the WNN. In conclusion, the performance of the WNN is better than that of the BPNN, which is more suitable for the evaluation of landscape ecological status.

RETRACTED

### 4.2. Error Analysis of the Landscape Ecological Evaluation Model

Using the previous sample data, this paper analyzes the evaluation error of the landscape ecological evaluation model based on the WNN. Eight sample data are selected, the landscape ecological evaluation model is used to evaluate these sample data, and the error between the output value of the model and the real value of the landscape ecological comprehensive evaluation index is compared, as shown in Figure 8.

As can be seen from Figure 8, the maximum error of the output value of the landscape ecological comprehensive evaluation model is 0.0010, the minimum error is 0.0006, the average error is 0.0053, and the accuracy is 0.001, which meets the actual demand. The above results show that the evaluation error of landscape ecological status based on the WNN is small, the accuracy of the model is high, and it has high practicability.

### 4.3. Accuracy of the Landscape Ecological Evaluation Model

The landscape ecological evaluation model is used to evaluate the sustainability of landscape land resources. The sustainability of landscape land resources can be divided into excellent sustainability (*V*1), outstanding sustainability (*V*2), high sustainability (*V*3), medium sustainability (*V*4), general sustainability (*V*5), and weak sustainability (*V*6). The corresponding scores are shown in Table 4.

In order to verify the evaluation accuracy of the landscape ecological evaluation model, 300 sample data were used to test it. The test results are shown in Table 5.

It can be seen from Table 5 that the accuracy rate of the landscape ecological evaluation model for *V*2, *V*4, and *V*5 is 100%, for *V*1 and *V*3 is 98%, and for *V*6 is 96%, and the overall accuracy rate is 98.67%. The above results show that the evaluation accuracy of the landscape ecological evaluation model is high, which can effectively evaluate the ecological status of the landscape and facilitate the ecological planning of the landscape.

## 5. Conclusion

Ecological planning of the landscape can improve the status of the ecological environment, ensure the good development of the ecological environment, and also make people feel the importance of environmental protection. This paper combines wavelet analysis and artificial neural network to build a wavelet neural network algorithm and builds a landscape ecological evaluation model based on wavelet neural network algorithm, so as to evaluate the ecological status of the landscape and provide data support for ecological planning of the landscape. The results show that the wavelet neural network needs 1700 training times to achieve the target accuracy, while the BP neural network needs 5300 training times, 3600 times more than the wavelet neural network. The MSE and MAE of the WNN were 5.3433 and 0.9829 times lower than those of the BP neural network, respectively. The MSE and MAE of the WNN were 5.0204 and 0.8764 times lower than those of the BP neural network, respectively. The accuracy of the model was 98.67%. The average error between the output value and the real value of the model was 0.0053, and the precision was 0.001. The above results show that the evaluation accuracy of the landscape ecological evaluation model is high, and the error is low, which can effectively evaluate the ecological status of the landscape and then facilitate the ecological planning of the landscape, and it has high practicability. The study does not take into account the impact of some small probability situations on landscape ecological planning, which needs to be further improved.

RETRACTED

## Figures and Tables

**Figure 1:** Evaluation process of the ecological status of the landscape based on the WNN model.

**Figure 2:** Mapping analysis of landscape ecology.

**Figure 3:** Evaluation index system of landscape ecological status.

**Figure 4:** Schematic diagram of the artificial neuron structure.

**Figure 5:** The structure of the BP neural network.

**Figure 6:** Structure of the wavelet neural network.

**Figure 7:** Comparison of training efficiency between the wavelet neural network and BP neural network.

**Figure 8:** Error between the output value and the real value of the model to the comprehensive evaluation index of landscape ecology.

**Table 1:** Comprehensive evaluation standard of landscape ecology.

Evaluation value	0–45	46–60	61–75	76–90	91–100
Corresponding level	Very poor	Poor	General	Good	Very good

**Table 2:** Evaluation error of the regional landscape ecological value.

Model	BPNN	WNN
MSE	5.4072	0.0639
MAE	1.1330	0.1501

**Table 3:** Landscape diversity assessment results of the landscape architecture.

Model	BPNN	WNN
MSE	5.0801	0.0597
MAE	0.9914	0.1150

**Table 4:** Sustainability classification of land resources.

Level	*V*1	*V*2	*V*3	*V*4	*V*5	*V*6
Score	90–100	80–89	70–79	60–69	50–59	0–49

**Table 5:** Test result.

Evaluation cycle	Rating					
Real quantity	*V*1	*V*2	*V*3	*V*4	*V*5	*V*6
Number of evaluations	50	50	50	50	50	50
Assessment accuracy	51	50	49	50	50	48
Evaluation cycle (%)	98	100	98	100	100	96

RETRACTED

## Data Availability

The data used to support the findings of this study are available from the corresponding author upon request.

## References

[1] Wang Y., Nan L., Zhang N. (2021). Application of Container building in community ecological environment renewal—taking gejiaying community in wuhan as an example. *IOP Conference Series: Earth and Environmental Science*.

[2] Xiao Y., Tian K., Huang H., Wang J., Zhou T. (2021). Coupling and coordination of socioeconomic and ecological environment in Wenchuan earthquake disaster areas: case study of severely affected counties in southwestern China. *Sustainable Cities and Society*.

[3] Wu J. (2019). Linking landscape, land system and design approaches to achieve sustainability. *Journal of Land Use Science*.

[4] Mander Ü., Kull A., Uuemaa E. (2018). Green and brown infrastructures support a landscape-level implementation of ecological engineering. *Ecological Engineering*.

[5] Peng K., Cao X., Liu B. (2021). Ensemble empirical mode decomposition with adaptive noise with convolution based gated recurrent neural network: a new deep learning model for South Asian high intensity forecasting. *Symmetry*.

[6] Dhibi N., Ben Amar C. (2021). Performance of genetic algorithm and levenberg marquardt method on multi-mother wavelet neural network training for 3D huge meshes deformation: a comparative study. *Neural Processing Letters*.

[7] Huang Y., Chao L. (2021). Accurate heating, ventilation and air conditioning system load prediction for residential buildings using improved ant colony optimization and wavelet neural network. *Journal of Building Engineering*.

[8] Alexander H., Ján P., Milan A., Jana M., Kamil Ž. (2020). Comparative study of week-ahead forecasting of daily gas consumption in buildings using regression ARMA/SARMA and genetic-algorithm-optimized regression wavelet neural network models. *Journal of Building Engineering*.

[9] Tang Y., Tang Y., Wu X., Chen H., Zeng T. (2020). Prediction of the antifreeze of the concrete structure based on random forest and wavelet neural network. *IOP Conference Series: Earth and Environmental Science*.

[10] Hasanzadeh Fereydooni R., Hassan S., Ali Shayanfar H., Houshang Mazinan A. (2020). sEMG-based variable impedance control of lower-limb rehabilitation robot using wavelet neural network and model reference adaptive control. *The Industrial Robot*.

[11] Xu M., Chu X., Fu Y., Wang C., Wu S. (2021). Improving the accuracy of soil organic carbon content prediction based on visible and near-infrared spectroscopy and machine learning. *Environmental Earth Sciences*.

[12] Du W., Zhang Q., Chen Y., Ye Z. (2021). An urban short-term traffic flow prediction model based on wavelet neural network with improved whale optimization algorithm. *Sustainable Cities and Society*.

RETRACTED

[13] Luo S., Lewis F. L., Song Y., Garrappa R. (2021). Dynamical analysis and accelerated optimal stabilization of the fractional-order self-sustained electromechanical seismograph system with fuzzy wavelet neural network. *Nonlinear Dynamics*.

[14] Dexu B., Weiwei K., Yunlong Q. (2019). A task-space tracking control approach for duct cleaning robot based on fuzzy wavelet neural network. *Journal of Dynamic Systems, Measurement, and Control*.

[15] Gaudin T. (2018). Investigating the impact of sugar-based surfactants structure on surface tension at critical micelle concentration with structure-property relationships. *Journal of Colloid and Interface Science*.

[16] Thi Yen V., Yao Nan W., Pham C. (2019). Recurrent fuzzy wavelet neural networks based on robust adaptive sliding mode control for industrial robot manipulators. *Neural Computing and Applications*.

[17] Mohammadzadeh A., Zhang W. (2019). Dynamic programming strategy based on a type-2 fuzzy wavelet neural network. *Nonlinear Dynamics*.

[18] Arthur C. K., Amoako Temeng V., Yao Y. Z. (2019). Soft computing-based technique as a predictive tool to estimate blast-induced ground vibration. *Journal of Sustainable Mining*.

[19] Lee Y., Lee T. W. (2019). Organic synapses for neuromorphic electronics: from brain-inspired computing to sensorimotor nervetronics. *Accounts of Chemical Research*.

[20] Bu D., Kong W., Qi Y. (2019). A task-space tracking control approach for duct cleaning robot based on fuzzy wavelet neural network. *Journal of Dynamic Systems, Measurement, and Control*.

[21] Han J.-X., Ma M.-Y., Wang K. (2021). Product modeling design based on genetic algorithm and BP neural network. *Neural Computing and Applications*.

[22] Najafzadeh M., Zeinolabedini M. (2018). Derivation of optimal equations for prediction of sewage sludge quantity using wavelet conjunction models: an environmental assessment. *Environmental Science and Pollution Research*.

[23] Zeinolabedini M., Najafzadeh M. (2019). Comparative study of different wavelet-based neural network models to predict sewage sludge quantity in wastewater treatment plant. *Environmental Monitoring and Assessment*.

